RETRACTED

# Knockdown of lncRNA ENST00000603829 Inhibits the Proliferation and Invasion of Salivary Gland Pleomorphic Adenoma through Regulating Cyclin D1

**DOI:** 10.1155/2022/8805305

**Published:** 2022-04-27

**Authors:** Yi Xu, Xin Sun, Jing Chen, Jinbiao Xu, Junshui Wei

**Affiliations:** Department of Stomatology, Taizhou First People's Hospital, Taizhou, Zhejiang 318020, China

## Abstract

**Objective:**

Salivary gland pleomorphic adenoma (SPA) is a benign neoplasm that can still recur even after radical surgery. To investigate its underlying pathogenesis, here, we examined the significance of lncRNA ENST00000603829 in the proliferation and invasion of SPA.

**Methods:**

SPA tissues (*n* = 30) and adjacent normal tissues (NC; *n* = 30) were collected from SPA patients treated at our hospital from June 2017 to December 2019. The human normal salivary gland epithelial cell line (HSG) and SPA cells (PA30, PA37, and PA116) were cultured. qRT-PCR was used for detecting the expression of cyclin D1 and lncRNA ENST00000603829 in tissues and cells. lncRNA ENST00000603829/cyclin D1 was knocked down or overexpressed in PA116 cells. The expression of cyclin D1 and lncRNA ENST00000603829 in different cell lines was examined using qRT-PCR. Transwell assays and cell counting kit-8 (CCK-8) were used to assess cellular invasion and proliferation. The testing result regarding the apoptosis rate and cell cycle was obtained via flow cytometry. Western blot provided the measurement of cyclin D1 expression in cells.

**Results:**

We observed an upregulation of lncRNA ENST00000603829 and cyclin D1 expression in SPA tissues and cells. Knockdown of lncRNA ENST00000603829 inhibited cell invasion and proliferation, promoting apoptosis and retaining the cells during the G0/G1 phase. However, such effects of lncRNA ENST00000603829 knockdown were inhibited when cyclin D1 was overexpressed.

**Conclusion:**

lncRNA ENST00000603829 can promote the occurrence and development of SPA through increasing cyclin D1 expression.

## 1. Introduction

Salivary gland pleomorphic adenoma (SPA) comprises of 40–70% of all salivary gland tumors [1]. In salivary gland tumors, the proportion of benign tumor is about 80%, while the malignant tumor merely occupies a small number [2]. Regarding the location, parotid tumors account for approximately 80% of this tumor, of which 40% belong to malignant tumor and the commonest kind belongs to PA [3, 4]. Histologically, SPA includes epithelial cells that form structures of the duct and modified myoepithelial cells (MEC) embedded in the chondromyxoid matrix [5]. It has been reported that adenomas originate from intercalated duct cells and MECs differentiate into epithelial and connective tissues [6]. SPA is benign and surgical excision is curative for it; however, there is a possibility of recurrence. Moreover, recurrent lesion grows rapidly with pain and nerve invasion [6–8] and even deteriorates into carcinoma ex-PA (Ca-ex-PA) with a possibility of metastasis and death [9]. As a result, the pathogenesis of SPA needs to be explored in depth to find scientific methods for treating the disease and preventing disease recurrence and progression.

RETRACTED

Cyclins have important roles in the development of PA. Further, studies have shown the possibility of an involvement of cell cycle markers cyclin D1, p-16, E2F, and CDK4 in PA's relapse and malignant transformation [10]. Some studies have used microarray analysis to investigate mRNAs and lncRNA expression in human SPA, and the performance of lncRNA-mRNA coexpression network analysis served to show the interaction of five key regulators (cyclin D1, CTNNB1, PLAG1, TP53, and IGF2) and multiple lncRNAs [11].

Studies have shown that in spite of the fact that from the human genome, many RNA species have been transcribed, the total transcripts include only a fraction of protein-coding sequences, with the remaining part being occupied by noncoding RNAs (ncRNAs) [12]. The latter can produce transcripts with functional small peptides and lack coding potential [12]. Accumulating evidence has highlighted that there is a possibility that ncRNAs are essential for cellular processes to develop into diseases [13]. Long ncRNAs (lncRNAs), which could be more than 200 nt, are involved in regulating epigenetic gene expression besides regulation of gene expression at the level of posttranscription and transcription [14]. The regulation method of lncRNAs includes histone modification, genetic imprinting, chromatin remodeling, transcriptional interference, transcriptional activation, cell cycle regulation, and nuclear transport [15, 16]. Yuan et al. provided evidence in their research that high levels of lncRNA-ATB led to notable promotion of the invasion-metastasis cascade of liver cancer [17]. Saito et al. confirmed increased levels of lncRNA-ATB in the tissues of gastric cancer as well as the existence of a close relationship between this lncRNA and vascular infiltration in addition to overall survival [18]. Jia et al. demonstrated that downregulating lncRNA-ATB led to metformin inhibiting the migration, invasion, and proliferation of VSMCs [19]. Also, as previously reported, many lncRNA transcripts that affect the pathogenesis of primary Sjögren's syndrome were dysregulated in this disease [20]. However, the association between lncRNAs and salivary gland diseases has not been studied extensively. Wei et al. revealed that in PA, lncRNA ENST00000603829 showing upregulated expression was associated with the key regulator CCND1 [21].

lncRNA ENST00000603829 is a newly discovered lncRNA of 541 nt in length, located on chr19: 58379338-58380202. However, its function and mechanism on PA have been reported minimally. This presents research attempts to investigate lncRNA ENST00000603829's mechanism and its effects on SPA cells through in vitro assays, aiming at finding new targets for the treatment of SPA, as well as at providing an effective experimental basis.

RETRACTED

## 2. Materials and Methods

### 2.1. Tissue Sample Collection

The tumor tissue (SPA; *n* = 30) and adjacent normal tissues (NC; *n* = 30) were obtained from SPA patients who were treated at Taizhou First People's Hospital during the period of time that starts in June 2017 and ends in December 2019. The identification of SPA tissues was made by three independent pathologists. The study protocol gained consent from the ethics committee of our hospital and strictly followed the Declaration of Helsinki. Informed consent was obtained from all patients for their participation in this research. This study was approved by the medical ethics committee of Taizhou First People's Hospital.

### 2.2. Cell Culture

The human normal salivary gland epithelial cell line (HSG) and SPA cells (PA30, PA37, and PA116) were provided by the American Type Culture Collection (ATCC). Culture of the entire cell lines was performed in Dulbecco's modified Eagle's medium (DMEM) containing 10 mg/mL streptomycin (Gibco, USA), 100 U/mL penicillin, and 10% fetal bovine serum (FBS) (Gibco, USA). Next, an incubator that was with 5% CO_2_ and was at the temperature of 37°C was then used for the purpose of culture.

### 2.3. Cell Transfection

Briefly, 6-well plates at a density of 2 × 10^5^ cells/well were used for cell transfection. Upon attaining cell confluence of 70–80%, using the Lipo 3000 Kit (Thermo, USA), the cells were transfected with negative siRNA plasmid (siNC), lncRNA ENST00000603829 siRNA plasmid (si-lncRNA ENST00000603829), negative pcDNA (pcNC), lncRNA ENST00000603829 pcDNA (pc-lncRNA ENST00000603829), and cyclin D1 pcDNA (cyclin D1). The media were replaced after transfection of 6 hours, and then, the cells were cultured for a further 48 hours and collected for subsequent experiments.

### 2.4. qRT-PCR

Tissues and cells were treated with the TRIzol method, which was performed to extract their total RNA. Subsequently, NanoDrop was used to examine total RNA's purity besides concentration and cDNA (Thermo, USA) was prepared according to the random primer reverse transcription kit. The expression levels of lncRNA ENST00000603829 and cyclin D1 mRNA were detected following the manufacturer's protocol of the SYBR GREEN Kit (TaKaRa, Japan), with GAPDH as the internal reference and 6 replicates of this experiment. The 2^−ΔΔ*Ct*^ method was employed for the purpose of calculating the target gene's relative expression.  Table 1 displayed the primer sequences as follows.

RETRACTED

### 2.5. Cell Counting Kit-8 (CCK-8)

First, 96-well plates were utilized for seeding the transfected PA116 cells (5 × 10^4^ cells) with 200 *μ*L fresh DMEM complete after 24 hours, 48 hours, and 72 hours of culture. Then, 10 *μ*L of CCK-8 detection solution was added to each well and cultured for 1.5 hours in an incubator, after which their absorbance was measured at 450 nm.

### 2.6. Cell Apoptosis

Cell apoptosis was measured by flow cytometry using Annexin V-FITC and 10 *μ*L of propidium iodide (PI) (20 mg/L) following the manufacturer's instructions. The apoptotic index was estimated using the following equation: apoptotic index = number of apoptotic cells/(number of apoptotic cells + number of normal cells) × 100%.

### 2.7. Cell Cycle

Briefly, transfected cells were trypsinized, washed twice with prechilled sterile PBS, fixed in 70% ethanol, and stained with 50 *μ*g/mL of PI. Then, the stained cells were analyzed by flow cytometry.

### 2.8. Transwell Assay

For this experiment, a Matrigel (BD Biosciences, USA) was inserted at the bottom of the upper chamber. Briefly, 100 *μ*L of cell suspension in serum-free media was added to the upper chamber, while 700 *μ*L of medium containing 10% FBS was added to the lower chamber. After 24 hours of incubation at 37°C with 5% CO_2_, the invaded cells were fixed with 4% paraformaldehyde and stained with 0.1% crystal violet solution. Lastly, images from 3 fields were randomly captured with an inverted microscope and the invaded cells were counted.

### 2.9. Western Blot

We first collected the cell lines and tissues for total protein extraction using cell lysate. Then, the supernatant proteins were collected after centrifugation at 12,000 rpm for 5 minutes at 4°C. Next, the BCA protein assay was used to determine the protein concentration. Subsequently, 20 *μ*g of protein with 1x loading buffer was boiled for denaturation. SDS-PAGE was then used for protein electrophoresis, and the proteins were transferred onto PVDF membranes. After one hour of blocking the membranes using 5% skim milk powder, the membranes were incubated with primary antibodies (cyclin D1 (ab134175, Abcam); CDK6 (ab124821, Abcam), and p21 (ab109520, Abcam)) overnight at a temperature of 4°C. Next, the membranes were washed thrice and incubated for one hour with secondary antibodies at ambient temperature, followed by three washing. The membranes were then developed using an enhanced chemiluminescence reagent, and the blots were detected using an enhanced chemiluminescence system. The ImageJ software was used to analyze the grayscale values of bands. GAPDH (ab8245, Abcam) was utilized as an internal reference for calculating the relative protein expression.

RETRACTED

### 2.10. Statistical Analysis

SPSS (version 24.0) was used for statistical analysis. The one-way analysis of variance was used for making comparisons among multiple groups, while the comparison between two groups was made by utilizing an independent *t*-test. The results of measurement data were expressed as mean ± standard deviation (SD). Pearson correlation analysis was performed to analyze the correlation between lncRNA ENST00000603829 and cyclin D1 expression in SPA tissues. *p* < 0.05 refers to a statistical difference.

## 3. Results

### 3.1. lncRNA ENST00000603829 Is Upregulated in SPA Tissues and Cells

We detected lncRNA ENST00000603829 expression in SPA. The results revealed a notable increase of lncRNA ENST00000603829 expression in SPA tissues compared to the normal ones (Figure 1(a)). Meanwhile, its expression in SPA cell lines was also notably increased compared with control HSG, with the highest expression in PA116 cells (Figure 1(b)).

### 3.2. Effect of lncRNA ENST00000603829 on the Growth Performance of SPA Cells

For the purpose of verifying the effect that lncRNA ENST00000603829 had on the growth performance of SPA cells, proliferation, invasion, apoptosis, and cell cycle of PA116 cells were examined after knockdown or overexpression of lncRNA ENST00000603829. The results showed a significant reduction in lncRNA ENST00000603829 expression after knockdown of this lncRNA, while showing an opposite trend after overexpression of this lncRNA (Figure 2(a)), indicating successful transfection. Silence of lncRNA ENST00000603829 resulted in significantly decreased cell proliferation and increased apoptotic rate, while its overexpression caused opposite changes (Figures 2(b) and 2(c)). There was a considerable increase in the proportion of cells in the G0/G1 phase and a decrease in the S phase in the si-lncRNA ENST00000603829 group, while pc-lncRNA ENST00000603829 contributed to opposite changes (Figure 2(d)); the former group was also related to downregulation of cell invasion (Figure 2(e)). In addition, knockdown of lncRNA ENST00000603829 markedly decreased the protein expression of cyclin D1 and CDK6 while prompting p21; overexpression of this lncRNA resulted in opposite changes (Figure 2(f)). Collectively, the outcome demonstrated the influence that lncRNA ENST00000603829 had on the growth performance of SPA cells.

RETRACTED

### 3.3. lncRNA ENST00000603829 Positively Regulates Cyclin D1 Expression

When exploring lncRNA ENST00000603829's mechanism, we found that mRNA and protein expression of cyclin D1 (a key factor of SPA) were notably increased in SPA tissues and cells (Figures 3(a)–3(c)). Subsequently, cyclin D1 expression was significantly downregulated in cells after knockdown of lncRNA ENST00000603829 while increasing after overexpression of lncRNA ENST00000603829 (Figure 3(d)). Pearson correlation analysis indicated a positive correlation between lncRNA ENST00000603829 and cyclin D1 in SPA tissues (Figure 3(e)). Thus, lncRNA ENST00000603829 might regulate cyclin D1 expression.

### 3.4. Upregulation of Cyclin D1 Reverses the Inhibitory Effect of lncRNA ENST00000603829 Knockdown on SPA

We further analyzed the role of cyclin D1 and lncRNA ENST00000603829 in SPA. Compared with the siNC group, si-lncRNA ENST00000603829 notably reduced the invasion and proliferation of cells and improved the apoptosis rate. Besides, the latter notably increased the percentage of cells in the G0/G1 phase while decreasing that in the S phase. CyclinD1 and CDK6 decreased considerably, and p21 increased after lncRNA ENST00000603829 knockdown. However, the effects were opposite after lncRNA ENST00000603829 overexpression (Figures 4(a)–4(f)). The mentioned results demonstrated that cyclin D1 could reverse the effects of lncRNA ENST00000603829 knockdown.

## 4. Discussion

SPA mainly attacks patients over 60 years old, with no difference in sex [22]. The occurrence of this disease can be found in both major and minor salivary glands [23]. Although SPA is characterized by phenotypic, biological, and clinical heterogeneity at a high level, clinically, the misdiagnosis rate for SPA is as high as 41.81% [24]. Therefore, there is an urgent need for new diagnostic biomarkers for SPA. Benefiting from the advancement and wide use of high-throughput sequencing technology, many studies have revealed that it is possible to take lncRNAs as diagnostic markers of most diseases. For instance, lncRNA MALAT1 was identified as a potential prognostic biomarker in addition to the therapeutic target for people who are at an early stage of lung cancer because of its stability and specificity and this lncRNA showed the existence of a higher expression in nonsmall cell lung cancer tissues in comparison with the expression in adjacent tissues [25]. If there is a notable increase in lncRNA H19 expression in lung cancer tissues [26] and plasma of patients, the lncRNA H19 is likely to act as a serological biomarker to clinically diagnose lung cancer [27]. However, only a few studies focused on lncRNA diagnostic markers for SPA. In our study, lncRNA ENST00000603829 was upregulated in SPA tissues and cells in this trial, indicating a potential diagnostic biomarker for SPA.

RETRACTED

The change of lncRNA expression is a medical sign of diseases but also affects a series of signal transmissions in cells, subsequently resulting in changes in cellular physiological functions as well as metabolic status. Some scholars believe that the function of lncRNAs to regulate signals affects the occurrence and development of diseases. Loss of lncRNA HOTAIR has the pivotal effect of not only inducing apoptosis but also regulating proliferation, invasion, and migration of cells in breast cancer [28]. Knockdown of lncRNA HULC inhibited the malignant progression of hepatocellular carcinoma [29], while overexpression of lncRNA HULC can promote the growth of hepatocellular carcinoma cells and increase the weight and formation rate of xenograft tumors [30]. There is evidence that the expression changes of lncRNA CCAT1 are related to EMT processes, migration, invasion, cell cycle, proliferation, and apoptosis in multiple cancers [31]. Our experiments also demonstrated that overexpression of lncRNA ENST00000603829 promoted proliferation and invasion and inhibited the apoptosis of SPA cells, as well as retained the cell cycle in the S phase. This means that upregulation of lncRNA ENST00000603829 is able to facilitate the development of cancer cells as well as subsequent cancer progression.

Cyclin D1, on the other hand, is considered to be a protein encoded by the CCND1 gene, acting as a significant regulator of cell cycle in addition to a prognostic and predictive factor for cancer. According to previous evidence, it is feasible to take cyclin D1 as a biomarker to forecast the prognosis of esophageal squamous cell carcinoma [32]. By analyzing human clinical tissues, the high expression of cyclin D1 is strongly linked to the cell proliferation of pancreatic cancer [33] and to the inhibition of proliferation and invasion of breast cancer [34]. It has also been pointed out that it is feasible for cyclin D1 to act as a target of aspirin against tamoxifen resistance in breast cancer [35]. Our study found that cyclin D1 could be involved in regulating the biological viability of SPA cells. Recent reports have confirmed that the expression of cyclin D1 is regulated by lncRNAs. For example, lncRNA HULC can upregulate cyclin D1 to accelerate the growth of human liver stem cells and this effect is achieved through the miR675-PKM2 pathway [36]. lncRNA ENST00000603829 was found to upregulate the expression of cyclin D1 in this study. Collectively, it can be seen that lncRNA ENST00000603829 in SPA exerts its biological function through regulating cyclin D1.

RETRACTED

## 5. Conclusion

In summary, lncRNA ENST00000603829 expression was found upregulated in SPA and affected the growth performance and development of SPA cells by positively regulating cyclin D1 expression. These results suggest lncRNA ENST00000603829 as a promising diagnostic biomarker and could be a therapeutic target for SPA.

## Figures and Tables

**Figure 1:** lncRNA ENST00000603829 expression in SPA tissues and cells. lncRNA ENST00000603829 expression in SPA (a) tissues (^∗∗^*p* < 0.01 vs. the NC group) and (b) cells (^∗∗^*p* < 0.01 vs. the HSG group) determined by qRT-PCR.

**Figure 2:** Effect of lncRNA ENST00000603829 on the growth performance of SPA cells. (a) qRT-PCR for expression of lncRNA ENST00000603829; (b) CCK-8 for examining the proliferation rate; (c, d) flow cytometry for testing the apoptosis rate (c) and cell cycle (d); (e) transwell assay for checking cell invasion; (f) Western blot assay for expression of cyclin D1, CDK6, and p21. ^∗∗^*p* < 0.01vs. the siNC group, ^##^*p* < 0.01 vs. the pcNC group.

**Figure 3:** Effect of lncRNA ENST00000603829 on cyclin D1 expression. qRT-PCR assay for the cyclin D1 mRNA level in SPA tissues; (b) Western blot assay for cyclin D1 protein expression in SPA tissues, ^∗∗^*p* < 0.01 vs. the NC group; (c) qRT-PCR assay for the cyclin D1 mRNA level in SPA cells, ^∗∗^*p* < 0.01 vs. the HSG group; (d) qRT-PCR assay for cyclin D1 mRNA levels in cells after overexpression or knockdown lncRNA ENST00000603829, ^∗∗^*p* < 0.01 vs. the siNC group, ^∗∗^*p* < 0.01 vs. the pcNC group; (e) Pearson correlation analysis of the correlation between lncRNA ENST00000603829 and cyclin D1 expression in SPA tissues.

**Figure 4:** Effect of cyclin D1 upregulation on tumor inhibition after knockdown of lncRNA ENST00000603829. qRT-PCR assay for cyclin D1 expression in cells; (b) CCK-8 assay to examine the cell proliferation rate; (c, d) flow cytometry was used for assessing the (c) cell apoptosis rate and (d) cell cycle; (e) transwell assay for invasion ability of cell; (f) Western blot assay for expression of cell cycle-related proteins (cyclin D1, CDK6, and p21). ^∗∗^*p* < 0.01 vs. the siNC group, ^##^*p* < 0.01 vs. the si-lncRNA ENST00000603829 + pcNC group.

**Table 1:** Primer sequences for qRT-PCR.

RNA	Sequences (5′ to 3′)
lncRNA ENST00000603829	F: 5′-TGAAGTAGGACTGGGCAGAGA
	R: 5′-TTTGGGTCAGGTGTCCACTC
Cyclin D1	F: 5′-TCTACACCGACAACTCCATCCG
	R: 5′-TCTGGCATTTTGGAGAGGAAGTG
GAPDH	F: 5′-GTCTCCTCTGACTTCAACAGCG
	R: 5′-ACCACCCTGTTGCTGTAGCCAA

## Data Availability

The data used to support the findings of this study are available from the corresponding author upon request.
